The article "Analysis of Microbiological and Clinical Characteristics of Bacterial Infection in Patients with Pulmonary Infection" was retracted in 2022. Reason: concerns about the peer review.

# Analysis of Microbiological and Clinical Characteristics of Bacterial Infection in Patients with Pulmonary Infection

**DOI:** 10.1155/2022/5607358

**Published:** 2022-06-16

**Authors:** Taimei Duan

**Affiliations:** The First People's Hospital of Chongqing Liangjiang New Area, Chongqing 401121, China

## Abstract

**Objective:**

Using data investigation, the microbiology of bacterial infection in patients with pulmonary infection was discussed, and its clinical characteristics were analyzed.

**Methods:**

The clinical data of 160 patients with pulmonary infection in our hospital from March 2019 to March 2021 were collected and analyzed. Blood samples were collected and cultured, and the pathogens were identified. The distribution, constituent ratio, and drug resistance of pathogens in elderly patients with pulmonary infection were analyzed. Logistics regression analysis was adopted to analyze the risk factors of pulmonary infection.

**Results:**

Of the 160 patients with pulmonary infection, 107 were males (66.88%) and 53 were females (33.13%). The age ranged from 12 to 97 years old, with an average of 63.82 ± 12.64 years old. Sevent-six patients (47.50%) were over 65 years old. Urban patients accounted for 71.88%, and rural patients accounted for 28.13%, of which workers accounted for 46.25%, and farmers and cadres each accounted for about 4%. 85.62% of smokers have smoked for more than 4 years. Eighty-five patients had chronic diseases such as coronary heart disease, hypertension, diabetes, and cerebrovascular disease. Heart failure occurred in 10.00%, old tuberculosis in 11.25%, and new tuberculosis in 5.63%. The average hospital stay of the patients was 14.93 days, and the improvement rate was 91.25%. Eleven patients died. Among the 160 patients with pulmonary infection, COPD, pneumonia, and lung cancer accounted for the highest proportions, and idiopathic pulmonary fibrosis, bronchitis dilatation, tuberculosis, and bronchial asthma also played an important role. Pathogenic bacteria were detected in 104 of the 160 elderly patients with pulmonary infection, and the detection rate was 65.00%. A total of 444 strains of pathogenic bacteria were detected, including 328 strains of Gram-negative bacteria (73.87%, mainly *Klebsiella pneumoniae*, *Pseudomonas aeruginosa*, *Stenotrophomonas maltophilia*, and *Serratia marcescens*), 28 strains of Gram-positive bacteria (6.30%, mainly *Staphylococcus aureus*), and 88 strains of fungi (20.00%, mainly *Candida albicans*). Regarding *Klebsiella pneumoniae* in elderly patients with pulmonary infection, the drug resistance rates were 59.72% for amoxicillin-clavulanate potassium, 52.78% for ampicillin sodium-sulbactam sodium, and 51.39% for cefazolin sodium. Regarding *Pseudomonas aeruginosa*, the drug resistance rates were 29.31% for ticarcillin sodium-potassium clavulanate, 27.59% for piperacillin sodium, and 24.14% for gentamicin. Regarding *Stenotrophomonas maltophilia,* the drug resistance rates were 79.55% for ceftazidime, 38.64% for chloramphenicol, and 31.82% for levofloxacin. Regarding *Serratia marcescens*, the drug resistance rates from high to low were 74.42% for cefotaxime, 72.09% for moxifloxacin, and 69.77% for gentamicin. Regarding *Staphylococcus aureus* in elderly patients with pulmonary infection, the drug resistance rates were 100.00% for penicillin, 61.54% for erythromycin, 61.54% for clarithromycin, and 61.54% for azithromycin. Regarding *Candida albicans*, the drug resistance rates from high to low were 22.41% for caspofungin, 15.52% for itraconazole, and 9.09% for fluconazole. The results of univariate analysis of pulmonary bacterial infection indicated that there were no significant differences in sex and body mass index between nonbacterial infection group and bacterial infection group (*P* > 0.05). There were significant differences in terms of dust or harmful gas exposure, family member smoking, chronic lung disease history, age, smoking, family cooking, hospital stay, and indwelling catheter (*P* < 0.05). Exposure to dust or harmful gases, family cooking, age, history of chronic lung disease, indwelling catheter, and length of hospital stay were risk factors for pulmonary bacterial infection (*P* < 0.05).

**Conclusion:**

Gram-negative bacteria are the main pathogens in elderly patients with pulmonary infection. Antibiotics should be administered reasonably according to the results of the drug sensitivity test. Older age, history of chronic lung disease, catheter indwelling, and length of stay are the risk factors for pulmonary bacterial infection.

## 1. Introduction

Pulmonary infection is a common respiratory disease in hospitalized patients [1]. Due to the abuse of hormones and the increase of antibiotic-resistant bacteria, coupled with the decline of patients' immunity, the incidence of pulmonary infection is increasing year by year. It brings great difficulties to the prevention and diagnosis and treatment of pulmonary infection in clinics [2]. The study found that, with the increase of age, the organ function of patients with pulmonary infection decreased more and more seriously, and the mortality rate showed an upward trend. At present, the specific pathogenesis of pulmonary infection is not completely clear [3]. The immune function of elderly patients is low, and the risk of pulmonary infection in patients with chronic respiratory diseases is significantly increased [4]. Feedback injury to the lungs leads to respiratory failure, which is life-threatening. It is found that pulmonary infection is secondary to other diseases, and the incidence of primary pulmonary infection is low, mainly bacterial infection.

Today, although we have entered the era of antibiotics, pulmonary infection still occupies an important position in respiratory diseases and is still one of the main diseases that threaten human health [5]. Infectious diseases account for about 1/3 of the global population deaths, among which acute respiratory infections account for 1/4. Statistics in the pharmaceutical industry show that 2/3 of the antibiotic prescriptions use dry respiratory tract infections, of which *β*-lactams, quinolones, and macrolides are the most adopted [6]. Therefore, this type of disease must be fully studied to achieve the purpose of reducing the mortality rate, hospitalization time, and medical expenses.

In the study of pulmonary infection, etiology plays the most direct and effective role in guiding clinical work, and it is also one of the most adopted and complex problems in clinics, which is concerned by clinicians [7]. Because the pathogens of pulmonary infection are complex and diverse, are closely related to the health status of the whole body and other organs, and are seriously disturbed by the normal flora of the environment and respiratory tract and some adaptive changes of pathogens to the living environment in recent years, newer and higher requirements have been put forward for etiological research, coupled with the recent continuous use of a wide variety of new antimicrobial agents, the application of immunosuppressants is increasing, and artificial channels are established [8]. Due to the application of mechanical channels, the number of refractory pulmonary infections increased significantly, the pathogens of infection were diversified, and drug-resistant bacteria increased significantly. Therefore, the drug resistance of pathogens and the application principles of antibiotics have changed accordingly, and empirical antibiotic treatment has encountered severe challenges.

For example, in 2004, the detection rates of *Staphylococcus aureus* and coagulase-negative staphylococci isolated from 14 hospitals in Shanghai accounted for 63.9% and 89.2%, respectively, compared with 62.7% and 76.9% in 2000. The resistance rates of *Pseudomonas aeruginosa* to ceftazidime and imipenem were more than 20% (24% and 21%, resp.).

The importance of etiological diagnosis of pulmonary infection has become increasingly prominent, especially in refractory and special pathogen infections [9]. However, “different grades of hospitals” in different regions have different types and habits of using antibiotics in the same hospital in different historical periods, and the distribution and degree of drug resistance of drug-resistant pathogenic bacteria are also very different, which is related to the size of the hospital, tge type of antimicrobial use, the length of time, the local economic level, and other factors [10]. For example, penicillin-resistant *Streptococcus pneumoniae* (PRSP) was 5% in 1987, 8% in 1992, and 25% in 1995 in the United States, 21% in Canada in 1994, and 48% in 1996. China's neighboring countries, such as Singapore (53%) and South Korea (89%), have a high incidence. PRSP in China is 13.9%∼42.7%, but 42.5∼83.6% of *Streptococcus pneumoniae* is resistant to erythromycin 4, which is much higher than 22.4%∼28.8% [11, 12] in Europe and the United States. Therefore, long-term monitoring of the spectrum of pathogenic bacteria and the law of drug resistance in this area, grasping its changing trend, issuing to clinical departments, and putting forward suggestions on the use of antibiotics, will help establish a perfect bacterial drug resistance monitoring system [13]. For clinicians' reference, it is of great significance to guide us to use antibiotics reasonably and accurately. Based on this, 160 cases of pulmonary infection treated in our hospital from March 2019 to March 2021 were discussed in this paper.

## 2. Patients and Methods

### 2.1. Normal Information

A total of 160 patients with pulmonary infection treated in our hospital from March 2019 to March 2021 were enrolled as the object of study. The clinical data were collected and analyzed. Blood samples were collected for culture, and pathogens were identified. The age of the patients was 18–83 years old, and the average age was 42.58 ± 20.83 years old. No statistical significance was shown in the comparison of general data of all patients. The Medical Ethics Association of our hospital approved the study, and informed consent was obtained from all patients.

Selection criteria were as follows: (1) regardless of gender, age ≥18 years old; (2) no cognitive, language, and intellectual impairment, with basic reading and writing ability; (3) meeting the diagnostic criteria of pulmonary infection in the guidelines for the diagnosis and treatment of community-acquired pneumonia in Chinese adults (2016 Edition); (4) the patient and/or his family members signed the relevant informed consent.

Exclusion criteria were as follows: (1) patients with severe heart, liver, renal insufficiency, malignant tumors, and other diseases; (2) old or pathological fractures; (3) refusing to participate; (4) patients with mental and psychological diseases.

### 2.2. Treatment Methods

The pathogenic bacteria were cultured with reference to the literature method [14]. The blood samples were inoculated on chocolate plates, blood plates and Sapaul medium (products of Shanghai Mérieux Company), and they were isolated and cultured for identification. Regarding the bacterial identification reference strains, *Staphylococcus aureus* ATCC25922, *Pseudomonas aeruginosa* ATCC27853, *Klebsiella pneumoniae* ATCC27644, *Escherichia coli* ATCC25923, *Acinetobacter baumannii* ATCC25934, and *Streptococcus pneumoniae* ATCC25948 were purchased from the American Type Biological Resource Collection Center.

### 2.3. Observation Index

Information such as smoking history, body mass index, home cooking time, hospitalization history, gender, age, and exposure to dust or harmful gases were recorded separately as indicators of observation.

### 2.4. Statistical Analysis

SPSS12.5 software was used for statistical analysis. The counting data are presented as [*n* (%)], and the chi-square test is used. Logistic regression analysis was adopted to analyze the influencing factors, and meaningful ones were included in the multi-factor logistic regression model. *P* < 0.05 indicates that the difference exhibits statistically significant.

## 3. Results

### 3.1. General Data Analysis of 160 Patients with Pulmonary Infection

First, we analyzed the general data of 160 patients with pulmonary infection who were admitted to our hospital from March 2019 to March 2021, including 107 males (66.88%) and 53 females (33.13%). The age range was from 12 to 97 years old, and the average age was 63.82 ± 12.64 years old. The age of 76 patients (47.50%) was over 65 years. Most of the patients came from urban areas (71.88%), while those from rural areas accounted for 28.13%, where the majority were workers (46.25%), and farmers and cadres each accounted for about 1/4. 85.62% of smokers have smoked more than 4 years. Of the 160 patients, 85 had chronic diseases such as coronary heart disease, hypertension, diabetes, and cerebrovascular diseases; 10.00% of had heart failure; 11.25% had old pulmonary tuberculosis; 5.63% had new tuberculosis. The average hospital stay of the patients was 14.93 days, and the improvement rate was 91.25%. Eleven patients died. All the results are indicated in Table 1.

### 3.2. Distribution of Pulmonary Diseases in 160 Patients

We analyzed the distribution of pulmonary diseases in 160 patients. COPD, pneumonia, and lung cancer accounted for the highest proportion, and idiopathic pulmonary interstitial fibrosis, bronchitis dilatation, tuberculosis, and bronchial asthma also played an important role. The specific results are indicated in Table 2.

### 3.3. Distribution and Constituent Ratio of Pathogens in 160 Elderly Patients with Pulmonary Infection

One hundred and four of 160 elderly patients with pulmonary infection had positive pathogens, with a detection rate of 65.00%. A total of 444 strains of pathogenic bacteria were detected, of which 328 strains (73.87%) were Gram-negative bacteria, including *Klebsiella pneumoniae, Pseudomonas aeruginosa, Stenotrophomonas maltophilia*, and *Serratia marcescens*. Twenty-eight strains of Gram-positive bacteria (6.30%, mainly staphylococci) and 88 strains of fungi (20.00%, of which *Candida albicans* were dominant). All the results are indicated in Figures 1–3.

### 3.4. Drug Resistance Rate of Gram-Negative Bacteria in Elderly Patients with Pulmonary Infection

We analyzed the drug resistance rate of Gram-negative bacteria in elderly patients with pulmonary infection. Regarding *Klebsiella pneumoniae* in elderly patients with pulmonary infection, the drug resistance rates were 59.72% for amoxicillin-clavulanate potassium, 52.78% for ampicillin sodium-sulbactam sodium, and 51.39% for cefazolin sodium. The resistance rates of *Pseudomonas aeruginosa* to ticarcillin sodium-potassium clavulanate, piperacillin sodium, and gentamicin were 29.31%, 27.59%, and 24.14%. The resistance rates of *Stenotrophomonas maltophilia* to ceftazidime, chloramphenicol, and levofloxacin were 79.55%, 38.64%, and 31.82%. Regarding *Serratia marcescens*, the drug resistance rates from high to low were 74.42% for cefotaxime, 72.09% for moxifloxacin, and 69.77% for gentamicin.. The specific results are indicated in Table 3.

### 3.5. Drug Resistance Rate of Gram-Positive Bacteria and Fungi in Elderly Patients with Pulmonary Infection

We analyzed the drug resistance rate of Gram-positive bacteria and fungi in elderly patients with pulmonary infection. Regarding *Staphylococcus aureus* in elderly patients with pulmonary infection, the drug resistance rates were 100.00% for penicillin, 61.54% for erythromycin, 61.54% for clarithromycin, and 61.54% for azithromycin. Regarding *Candida albicans*, the drug resistance rates from high to low were 22.41% for caspofungin, 15.52% for itraconazole, and 9.09% for fluconazole. The specific results are indicated in Tables 4 and 5.

### 3.6. Univariate Analysis of Pulmonary Bacterial Infection

We analyzed the single factor of pulmonary bacterial infection. One hundred and four cases of pathogens were detected in 160 patients with pulmonary infection as bacterial infection group, and the rest were nonbacterial infection group. No significant difference was found in sex and body mass index between nonbacterial infection group and bacterial infection group (*P* > 0.05), but there were significant differences in smoking, household cooking, exposure to dust or harmful gases, family smoking history, hospitalization time for chronic lung disease, and age of indwelling catheter (*P* < 0.05). The specific results are indicated in Table 6.

## 4. Discussion

With the aging population, the extensive use of broad-spectrum antibiotics, glucocorticoids, and the continuous emergence of immunosuppressive hosts such as organ transplantation and complex and refractory pulmonary infections are obviously on the rise, and the pathogens of infection are diversified and complicated [15]. The number of drug-resistant bacteria has increased remarkably, and the treatment of empirical antibiotics has been severely challenged. Therefore, the etiological diagnosis of pulmonary infection is very important. However, etiology usually takes a day to show results, so initial antimicrobial therapy is usually empirical. This requires us to carefully study and analyze the etiology of pulmonary infection to provide a basis for empirical treatment.

The habits and types of using antibiotics in different regions, different levels of hospitals, and different periods of the same hospital are different, and the distribution and degree of drug-resistant pathogenic bacteria are also very different [16]. This is related to the size of the hospital, the type of use of antibiotics, the length of time, the local economic level, and other factors [15, 16]. Therefore, monitoring the changes of common pathogenic bacteria and the changes of drug resistance is of special significance to guide the local clinical drug use.

In this group, there were 107 males (66.88%) and 53 females (33.13%). The age range was from 12 to 97 years old, and the average age is 63.82 ± 12.64 years old. 47.50% were over 65 years old, which caught our attention [17]. According to statistics, China is already a society with an aging population. It is estimated that by the middle of the century, the number of people over 65 years old will reach 322 million, accounting for 21.8% of the total population. The aging of society is increasingly becoming a social problem of great concern. Due to the pathophysiological characteristics of the elderly, the chest X-ray films of pulmonary infection may be missed and misdiagnosed, and their clinical manifestations, signs, and laboratory tests are often atypical [17, 18]. Difficult clinical diagnosis and treatment, poor prognosis, and high mortality have always been major problems affecting the health and life of the elderly.

In this group, up to 160 patients with coronary heart disease, hypertension, diabetes, cerebrovascular disease, and other chronic diseases are related to the high proportion of elderly cases. For elderly patients, the disease is often accompanied by aging. In the elderly, the reserve function of various organs is reduced or lost, the response to stress decreases, and the disease of one organ may lead to damage to another organ. For example, long-term bed rest or coughing in patients with cerebrovascular disease can easily lead to aspiration pneumonia, heart failure, which is closely related to pulmonary infection, and the probability of pulmonary infection in patients with diabetes increases. We should attach great importance to the previously mentioned situation.

The symptoms of pulmonary infection in the elderly are often not obvious, which increases the difficulty of clinical diagnosis, so laboratory examination is of great significance for the diagnosis and treatment of pulmonary infection in the elderly [19]. Extensive use of broad-spectrum antibiotics can cause severe bacterial resistance and increase the difficulty of clinical treatment of pulmonary infections in the elderly. Sputum culture and drug susceptibility testing of elderly patients with pulmonary infection can guide the use of antibiotics, reduce the incidence of bacterial resistance, and improve the cure rate.

Gram-negative bacilli were the main pathogens of pulmonary infection in inpatients. Some data indicates that it is 70%∼90% [2, 20]. Gram-negative bacteria accounted for 73.87% in this group, which was consistent with the conclusions of previous studies. Among all Gram-negative bacteria, *Pseudomonas aeruginosa* was the most common, followed by *Acinetobacter baumannii*, *Escherichia coli*, *Klebsiella pneumoniae*, *Stenotrophomonas maltophilia*, and *Haemophilus influenzae*. In this group of data, there are 28 strains of Gram-positive bacteria, accounting for 6.30% of the bacteria in this group, mainly staphylococci and enterococci [21]. Due to the wide use of various antimicrobials, hormones, and immunosuppressants, the problem of bacterial drug resistance is becoming more serious. The outbreak caused by drug-resistant bacterial infection is also increasing, and even many bacteria have MDR, which brings great difficulties to clinical treatment. Through the drug sensitivity statistics of different centers, it was found that the sensitivity of cefepime to strains from different regions was quite different. According to a multicenter nosocomial infection surveillance network in Belgium, 716 strains of *Pseudomonas aeruginosa* were studied [22]. A total of 50.5% of the strains were sensitive to cefepime and 29.5% were resistant, while the results of our study indicated that 74.3% were sensitive and 12.9% were resistant. According to foreign reports, sulbactam maintained good antibacterial activity against imipenem-resistant Acinetobacter in vivo and in vitro [23]. From 1995 to 1997, Corbell et al. treated 42 cases of *Acinetobacter baumannii* infection with sulbactam (18 cases) and amoxicillin-sulbactam (24 cases), and 39 cases were cured [24].

Anti-infective therapy is the most important treatment for pulmonary infection in the elderly. As most of the elderly are complicated with multiple underlying diseases, with concealed onset, rapid progress, and high mortality, empirical anti-infective treatment should be administered as soon as possible once pulmonary infection is diagnosed [25]. The choice of anti-infective regimens is critical, and studies by Alvarez et al. show that about 44% of patients need to adjust their anti-infective regimens after initial empirical anti-infective therapy, of which 62% are multidrug resistant bacterial infections [26]. Most of the elderly are prone to drug-resistant bacterial infection due to repeated hospitalization, long hospitalization time, and low immunity [27]. Therefore, in the selection of anti-infective drugs, only the third generation cephalosporins, quinolones, and *β*-lactamase inhibitors can be administered in noncritically ill patients without the risk of multiple drug resistance MDR. For noncritically ill patients with MDR risk, *β*-lactamase inhibitors against *Pseudomonas aeruginosa*, cephalosporins, and carbapenem can be administered [28]. For critically ill patients, the previously mentioned antibiotics can be adopted in combination with quinolone or aminoglycoside antibiotics against *Pseudomonas aeruginosa*. For patients at risk for MRSA, a combination of glycopeptides or linezolid can be used. Tigecycline or polymyxin can be adopted in patients at risk of infection with pan-resistant bacteria (susceptible only to classes 1 or 2 antibiotics) [29]. When the results of etiological examination and drug sensitivity come out, the anti-infection scheme can be further adjusted according to the results of drug sensitivity if necessary. According to the pharmacokinetics of the elderly due to the decline of liver and kidney function, the increase of adipose tissue, low albumin, and other reasons, the selection of antibiotic dose needs to adjust the dosage and times to optimize the antibacterial efficacy.

In this study, drugs with a high resistance to *Klebsiella pneumoniae* in elderly patients with pulmonary infection were amoxicillin-clavulanate potassium, ampicillin sodium-sulbactam sodium, and cefazolin sodium [30]. *Pseudomonas aeruginosa* had a high resistance rate to ticarcillin sodium-potassium clavulanate, piperacillin sodium, and gentamicin and were sensitive to Amikacin, polymyxin E, and polymyxin B. They were resistant to other antibiotics. *Stenotrophomonas maltophilia* had a high resistance rate to ceftazidime, chloramphenicol, and levofloxacin and were sensitive to compound sulfamethoxazole and minocycline. *Serratia marcescens* had a high resistance rate to cefotaxime, moxifloxacin, and gentamicin and were sensitive to piperacillin sodium-tazobactam sodium, cefoperazone sodium-sulbactam sodium, and ceftazidime [31]. Staphylococcus aureus had a high resistance rate to penicillin, erythromycin, clarithromycin, and azithromycin and were sensitive to doxycycline and vancomycin. Drugs with high resistance rates to *Candida albicans* from high to low were caspofungin, itraconazole, and fluconazole, and they were more sensitive to flucytosine, amphotericin B, and voriconazole. When selecting antibiotics in the clinical treatment of elderly patients with pulmonary infection, we should pay attention to the results of drug sensitivity test and adjust the use of drugs in time.

Recently, great attention has been paid to the risk factors of pulmonary bacterial infection in inpatients [32]. Epidemiology found that about 30.2% of hospitalized patients with pulmonary infection were related to their own conditions, such as physique, living habits, and medical history, and about 10.7% of hospitalized patients were related to clinical treatment. This study showed that age, chronic lung history, indwelling catheter, and length of stay were the risk factors of bacterial infection in pulmonary infection (*P* < 0.05). The infection rate of bacteria in the lungs of hospitalized patients who often cook at home and often encounter dust or harmful gases is also higher, mainly because there are more harmful substances in the kitchen, such as carbon monoxide, nitrogen, and sulfur oxides. These are all pathogenic factors that cause respiratory diseases. In addition, from the results of this study, catheter indwelling and length of stay in hospital are also closely related to pulmonary infection, which may be because longer hospital stays and catheter indwelling will increase patients' contact with pathogens, thus increasing the risk of bacterial infection.

Conclusively, *Klebsiella pneumoniae* is the main pathogen of pulmonary bacterial infection in inpatients in our hospital. Older age, history of chronic lung disease, exposure to dust or harmful gases, family cooking, long indwelling catheter, and long hospital stay are the risk factors of *Klebsiella pneumoniae* in patients staying at our hospital. Actively controlling the primary disease and increasing the frequency of lung detection can reduce the incidence and reduce the bacterial infection of the lung.

## Figures and Tables

**Figure 1:** Distribution and constituent ratio of Gram-positive bacteria.

**Figure 2:** Distribution and constituent ratio of Gram-negative bacteria.

**Figure 3:** Distribution and composition of fungi.

**Table 1:** General data of 160 patients with pulmonary infection [*n*/%].

General situation	Number of cases	Constituent ratio (%)
Gender		
Male	107	66.88
Female	53	33.13
Age (years)		
13∼44	23	14.38
45∼64	61	38.13
≥65	76	47.50
Body weight (kg)	63.82 ± 12.64	
Course of disease (year)	0.53 ± 0.18	
Number of smoking		
≥800 years' expenditure	24	15.00
600–799ears' expenditure	12	7.50
400–599ears' expenditure	18	11.25
<400ears' expenditure	23	14.38
Profession		
Farmers	40	25.00
Workers	74	46.25
Cadre	41	25.63
Students	5	3.13
Home place		
City	115	71.88
Rural areas	45	28.12
Diabetes	16	10.00
Coronary artery disease	24	15.00
Cerebral vascular disease	11	6.88
High blood pressure	34	21.25
Cardiac function (NYHA)		
0	144	90.00
1	1	0.63
2	5	3.13
3	8	5.00
4	3	1.88
Tuberculosis		
Obsolete	18	11.25
Newly found	9	5.63
Hospitalization days		
1–4	6	3.75
5–9	39	24.38
10–14	47	29.38
15–19	31	19.38
20–24	18	11.25
25–29	8	5.00
>30	10	6.25
Turn to		
Turn for the better	146	91.25
Pass away	11	6.88
Automatic discharge	1	0.63
Other	2	1.25

**Table 2:** Distribution of pulmonary diseases in 160 patients.

Disease type	Number of cases	Constituent ratio (%)
COPD	41	25.63
Pneumonia	38	23.75
Lung cancer complicated with infection	21	13.13
Idiopathic pulmonary interstitial fibrosis	12	7.50
Bronchiectasis	12	7.50
Bronchial asthma	7	4.38
Pulmonary tuberculosis	7	4.38
Acute bronchitis	5	3.13
Pleural effusion	3	1.88
Tuberculous pleurisy	2	1.25
Pulmonary cyst	2	1.25
Lung abscess	1	0.63
FOU	1	0.63
Empyema	1	0.63
Cryptogenic organic pneumonia	1	0.63
Pulmonary thromboembolism complicated with infection	1	0.63
Spontaneous pneumothorax	1	0.63

**Table 3:** Antimicrobial resistance of Gram-negative bacteria in 160 elderly patients with pulmonary infection.

Antibacterials	*Klebsiella pneumoniae* (*n* = 72)		*Pseudomonas aeruginosa* (*n* *=* 58)		*Stenotrophomonas maltophilia* (*n* = 44)		*Serratia marcescens* (*n* = 43)	
	Number Of plants	Drug resistance rate (%)	Number of plants	Drug resistance rate (%)	Number of plants	Drug resistance rate (%)	Number of plants	Drug resistance rate (%)

Amoxicillin-clavulanate potassium	43	59.72	—	—	—	—	—	—
Ampicillin sodium-sulbactam sodium	38	52.78	—	—	—	—	—	—
Cefazolin sodium	37	51.39	—	—	—	—	—	—
Ticarcillin sodium-clavulanate potassium	34	47.22	17	29.31	6	13.64	22	51.16
Chloramphenicol	29	40.28	—	—	17	38.64	25	58.14
Compound sulfamethoxazole	27	37.50	—	—	0	0	1	2.33
Moxifloxacin	26	36.11	—	—	—	—	31	72.09
Cefotaxime	24	33.33	—	—	—	—	32	74.42
Cefuroxime	24	33.33	—	—	—	—	—	—
Ciprofloxacin	20	27.78	6	10.34	—	—	23	53.49
Gentamicin	17	23.61	14	24.14	—	—	30	69.77
Tobramycin	14	19.44	10	17.24	—	—	20	46.51
Aztreonam	12	16.67	3	5.17	—	—	6	13.95
Cefepime	12	16.67	3	5.17	—	—	29	67.44
Piperacillin sodium-tazobactam sodium	11	15.28	9	15.52	—	—	0	0
Cefoperazone sodium-sulbactam sodium	9	12.50	6	10.34	6	13.64	0	0
Ceftazidime	9	12.50	6	10.34	35	79.55	0	0
Cefoxitin	9	12.50	—	—	—	—	—	—
Minocycline	9	12.50	—	—	0	0	0	0
Amikacin	6	8.33	0	0	—	—	2	4.65
Levofloxacin	6	8.33	7	12.07	14	31.82	20	46.51
Imipenem	0	0	1	1.72	—	—	0	0
Meropenem	0	0	1	1.72	—	—	0	0
Ertapenem	0	0	—	—	—	—	1	2.33
Tigecycline	0	0	—	—	—	—	0	0
Polymyxin E	—	—	0	0	—	—	—	—
Polymyxin B	—	—	0	0	—	—	—	—
Piperacillin sodium	—	—	16	27.59	—	—	—	—

**Table 4:** Antimicrobial resistance of 13 strains of *Staphylococcus aureus* in 160 elderly patients with pulmonary infection.

Antibacterials	Number of drug-resistant plants	Drug resistance rate (%)
Penicillin	13	100.00
Erythromycin	8	61.54
Clarithromycin	8	61.54
Azithromycin	8	61.54
Clindamycin	6	46.15
Gentamicin	3	23.08
Oxacillin	2	15.38
Levofloxacin	2	15.38
Ciprofloxacin	2	15.38
Tobramycin	2	15.38
Recurrent sulfamethoxazole	1	7.69
Rifampicin	1	7.69
Tetracycline	1	7.69
Moxifloxacin	1	7.69
Tigecycline	1	7.69
Amikacin	1	7.69
Doxycycline	0	0
Vancomycin	0	0
Linezolid	0	0
Minocycline	0	0
Chloramphenicol	0	0
Teicoplanin	0	0

**Table 5:** Antimicrobial resistance of 58 strains of Candida albicans in 160 elderly patients with pulmonary infection.Antibacterials.

	Number of drug-resistant plants	Drug resistance rate (%)
Caspofungin	13	22.41
Itraconazole	9	15.52
Fluconazole	5	8.62
Fluorocytosine	0	0
Amphotericin B	0	0
Voriconazole	0	0

**Table 6:** Single factor analysis of pulmonary infection.Influencing factors.

	Bacterial infection (*n* = 104)	Constituent ratio (%)	Nonbacterial infection (*n* = 56)	Constituent ratio (%)	*t*/*x*^2^	*P*
Gender						
Male	57	54.81	31	55.36	0.004	>0.05
Female	47	45.19	25	44.64		
Age (years)						
<18	27	25.96	6	10.71	9.675	<0.05
18–60	39	37.50	16	28.57		
>60	38	36.54	34	60.71		
Smoking						
Suction	27	25.96	49	87.50	55.277	<0.05
Do not suck	77	74.04	7	12.50		
Body mass index (kg/m^2^)						
<18.5	20	19.23	11	19.64	0.005	>0.05
18.5∼24.0	73	70.19	39	69.64		
>24.0	11	10.58	6	10.71		
Home cooking						
Yes	54	51.92	39	69.64	4.696	<0.05
No	50	48.08	17	30.36		
Exposure to dust or harmful gases						
Yes	9	8.65	14	25.00	7.902	<0.05
No	95	91.35	42	75.00		
Family members smoke						
Yes	55	52.88	39	69.64	13.908	<0.05
No	49	47.12	17	30.36		
History of chronic lung disease						
Yes	9	8.65	23	41.07	23.908	<0.05
No	95	91.35	33	58.93		
Length of stay (days)						
≤7	57	54.81	14	25.00	13.908	<0.05
>7	47	45.19	43	76.79		
Catheter indwelling						
Yes	41	39.42	43	76.79	20.376	<0.05
None	63	60.58	13	23.21		

## Data Availability

No data were used to support this study.
